# The Role of Deep Learning-Based Echocardiography in the Diagnosis and Evaluation of the Effects of Routine Anti-Heart-Failure Western Medicines in Elderly Patients with Acute Left Heart Failure

**DOI:** 10.1155/2021/4845792

**Published:** 2021-08-09

**Authors:** Jinyou Chen, Yue Gao

**Affiliations:** Department of General Practice, Affiliated Hangzhou First People's Hospital, Zhejiang University School of Medicine, Hangzhou 310000, Zhejiang, China

## Abstract

**Objective:**

The role of deep learning-based echocardiography in the diagnosis and evaluation of the effects of routine anti-heart-failure Western medicines was investigated in elderly patients with acute left heart failure (ALHF).

**Methods:**

A total of 80 elderly patients with ALHF admitted to Affiliated Hangzhou First People's Hospital from August 2017 to February 2019 were selected as the research objects, and they were divided randomly into a control group and an observation group, with 40 cases in each group. Then, a deep convolutional neural network (DCNN) algorithm model was established, and image preprocessing was carried out. The binarized threshold segmentation was used for denoising, and the image was for illumination processing to balance the overall brightness of the image and increase the usable data of the model, so as to reduce the interference of subsequent feature extraction. Finally, the detailed module of deep convolutional layer network algorithm was realized. Besides, the patients from the control group were given routine echocardiography, and the observation group underwent echocardiography based on deep learning algorithm. Moreover, the hospitalization status of patients from the two groups was observed and recorded, including mortality rate, rehospitalization rate, average length of hospitalization, and hospitalization expenses. The diagnostic accuracy of the two examination methods was compared, and the electrocardiogram (ECG) and echocardiographic parameters as well as patients' quality of life were recorded in both groups at the basic state and 5 months after drug treatment.

**Results:**

After comparison, the rehospitalization rate and mortality rate of the observation group were lower than the rates of the control group, but the diagnostic accuracy was higher than that of the control group. However, the difference between the two groups of patients was not statistically marked (*P* > 0.05). The length and expenses of hospitalization of the observation group were both less than those of the control group. The specificity, sensitivity, and accuracy of the examination methods in the observation group were higher than those of the control group, and the differences were statistically marked (*P* < 0.05). There was a statistically great difference between the interventricular delay (IVD) of the echocardiographic parameters of patients from the two groups at the basic state and the left ventricular electromechanical delay (LVEMD) parameter values after 5 months of treatment (*P* < 0.05), but there was no significant difference in the other parameters. After treatment, the quality of life of patients from the two groups was improved, while the observation group was more marked than the control group (*P* < 0.05).

**Conclusion:**

Echocardiography based on deep learning algorithm had high diagnostic accuracy and could reduce the possibility of cardiovascular events in patients with heart failure, so as to decrease the mortality rate and diagnosis and treatment costs. Moreover, it had an obvious diagnostic effect, which was conducive to the timely detection and treatment of clinical diseases.

## 1. Introduction

ALHF is a clinical syndrome such as ischemia, hypoxia, and dyspnea mainly resulting in pulmonary circulation congestion, which is caused by decreased acute myocardial contraction, increased left ventricular end-diastolic pressure, and decreased cardiac output due to valvular heart disease, myocardial damage, arrhythmia, and left ventricle overload [1]. The main clinical manifestation of the patient is acute pulmonary edema, which can lead to cardiogenic shock or cardiac arrest, which seriously threatens the patient's life safety [2]. According to relevant statistics, the mortality rate of elderly patients with ALHF is about 2.8% and the mortality rate within 3 months can be as high as 9.27%. Besides, half of them will be hospitalized again within half a year, so ALHF causes greater damage to the patient's body, and effective control can only be achieved by following the doctor's advice and timely treatment [3, 4]. Drug therapy is the most routine method of treatment, and the current clinical drugs include digitalis preparations, vasodilators, and diuretics. The patients with different causes or incentives are given different drug treatments, thus achieving effective therapeutic effects [5].

Echocardiography is to measure the periodic activities of the heart wall, ventricle, valve, and other structures underneath the chest wall and soft tissue by applying the principle of ultrasonic distance measurement pulsed ultrasound. Then, the measured results are presented on the display by the relationship curve between the corresponding activities and time of each structure, that is, the way of recording these curves with a recorder [6–8]. At present, it has been clinically applied in the monitoring of heart and large vessel structure, detection of blood flow velocity and type, esophagus, intravascular ultrasound, and evaluation of local myocardial perfusion [9–11].

In recent years, artificial intelligence has been widely adopted. By the 1990s, machine learning-related technologies such as supervised learning technology began to be applied to the processing of medical images. Medical images are input for training, useful features are extracted, and further operations such as classification are carried out. The introduction of this kind of method has realized the transformation of the medical image processing system from completely manual design and operation to a series of processing by the computer according to the designed algorithm to the input picture, saving a lot of human resources. Deep learning algorithm has also been introduced into the field of imaging, which can systematically standardize images or sounds by learning the internal laws and representation levels of sample data to improve the recognizability of imaging [12–14]. Among them, the DCNN algorithm has better application recognition performance in large-scale natural image data sets. This is mainly due to the use of a large amount of annotation data in deep learning, starting from the original pixels of the image, and layer-by-layer hierarchical learning. In this study, 80 elderly patients with ALHF were selected and treated with routine anti-left-heart-failure Western medicine. Then, echocardiography based on the DCNN learning algorithm was adopted, aiming to obtain objective images through automatic recognition and noise reduction sharpening processing of the algorithm, so as to diagnose and evaluate the effect of drug treatment on patients.

## 2. Materials and Methods

### 2.1. General Data

A total of 80 elderly patients with ALHF admitted to Affiliated Hangzhou First People's Hospital from August 2017 to February 2019 were selected as the research objects, and they were grouped randomly into the control group (*n* = 40) and the observation group (*n* = 40). There were 26 males and 14 females in the control group, aged 66–77 years, with an average age of 69.02 ± 1.24 years; arterial partial pressure of oxygen (PaO_2_) was 63.4 ± 16.3 mmHg, arterial partial pressure of carbon dioxide (PaCO_2_) was 38.5 ± 20.7 mmHg, and left ventricular ejection fraction (LVEF) was 46.3 ± 12.4%; there were 16 cases of grade II, 14 cases of grade III, and 10 cases of grade IV based on the heart function classification. The observation group was composed of 25 males and 15 females, and they were 65–76 years old, with an average age of 69.31 ± 1.36 years; PaO_2_ was 62.9 ± 16.2 mmHg, PaCO_2_ was 38.7 ± 19.8 mmHg, and LVEF was 47.4 ± 13.5%; there were 17 cases of grade II, 14 cases of grade III, and 9 cases of grade IV based on the heart function classification. Gold standards of diagnosis were as follows. The patient was diagnosed according to clinical manifestation, it was generally on the basis of the original heart disease, and the original symptoms were progressively aggravated. What is more, chest tightness, shortness of breath, palpitations, and paroxysm of dyspnea were aggravated at night. The patient sat breathing but could not lie supine. In combination with right heart failure, the patient could have anorexia, abdominal distension, edema of lower limbs, hepatosplenomegaly, etc., with heart color ultrasound examination and blood test.

Diagnostic criteria were referred to the relevant diagnostic criteria for ALHF in *Diagnosis and Treatment of Heart Failure*. The criteria for inclusion were defined to include patients who met the above diagnostic criteria, suffered from basic diseases such as coronary atherosclerotic heart disease or hypertension, clinically showed typical symptoms of heart failure, were not allergic to the therapeutic drugs or related preparations used in the echocardiogram examination in this study, and were aware of and signed the informed consent forms by themselves and their family members. The criteria for exclusion were defined to include patients who were combined with cognitive impairment, had poor compliance, were unable to cooperate with this research, were accompanied with abnormal liver and kidney function or in a state of stress, had pulmonary heart disease, and changed to other anti-heart-failure treatment methods in the course of this study.

### 2.2. Methods

#### 2.2.1. Deep Convolutional Neural Network Learning Algorithm

*(1) Basic Principles of Deep Convolutional Neural Network*. DCNN is continuously adjusted and optimized on the basis of the traditional neural network [15]. It retains the similar hierarchical structure of the neural network but has more layers. What is more, the processing performed by each layer is different, and the connection has also been simplified.

Under normal circumstances, the main components of a DCNN include data input layer, convolution layer, activation function, other processing layers, and output layer.

Most importantly, the input layer is responsible for receiving input data. Usually, the input layer is multidimensional and can retain the structural information of the data itself in the image. The convolutional layer uses the convolution kernel to operate and extract features from the input samples [16, 17]. Usually, the convolution kernel can change with the depth in the network. After convolution, basic information is extracted, such as lines and contours, and this information is determined by the position of the convolutional layer in the network; that is, the deeper the convolutional layer, the larger the receptive field. Therefore, the more local features considered by fusion, the more abstract features are extracted. The specific operation is as follows.

First, the characteristics of noise are counted, and the noise approximate model is shown in

(1) $$\begin{array}{c} yl=yl-1◎xl+jl. \end{array}$$

Here, *yl* − 1 represents the input of the l^th^ layer, ◎ stands for the convolution operation, *xl* means the number of convolutional layers, and *jl* indicates the bias. Finally, the extracted feature map *yl* is the output of the *l*^th^ layer.

The activation function is a critical part of DCNN, which can introduce nonlinear operations into the entire model. If there is no activation function, other linear operation layers are added to increase the depth of the network, which will make the expressive power of the entire network worse. Different activation functions will get different gradient derivatives when the network is backpropagated. In the development of deep learning networks, the specific operations are presented in equations (2)–(4) and Figure 1:

(2) $$\begin{array}{c} y=\frac{1}{\left(1+e-x\right)}, \end{array}$$

(3) $$\begin{array}{c} \tan\;h\left(x\right)=\frac{\left(1-e-2x\right)}{\left(1+e-2x\right)}, \end{array}$$

(4) $$\begin{array}{c} y=\left\{\begin{array}{cc} x, & x\geq 0,\\ 0, & x＜0. \end{array}\right) \end{array}$$

Pooling is used for local pooling operation on the feature map, which can remove part of the redundant information, shrink the feature map, reduce the amount of calculation, and maintain the position of the feature in the image. Moreover, it can also help the model to prevent overfitting [18, 19]. The existing general pooling operation window areas do not overlap, such as the commonly used average pooling and maximum pooling. Overlapping pooling means that the areas of adjacent pooling operations will overlap. There is also pyramid pooling, which can pool image convolution features of any scale into the same dimension.

In the full connection layer, each node is connected with all the nodes of the upper layer, which is adopted to synthesize the features extracted from the previous layer and output them to the output layer. Due to its fully connected nature, the fully connected layer generally has the largest number of parameters.

The output layer often uses Softmax to convert the direct processing output from the full connection into the probability distribution value of each class, and then, the class corresponding to the largest probability is selected as the sample classification for output [20, 21].

In the whole training process, the loss of this round is calculated based on the loss function after the input of the previous forward propagation through all levels and processing, and the backward propagation loss is propagated. Then, the parameters of each layer are updated in the direction of reducing the loss by using appropriate optimization methods such as stochastic gradient descent. Therefore, the loss function can be said to be the instructor of the entire network learning, which has a great influence on the quality of the final learning result. The existing commonly used loss function (mean square error loss function) can be expressed as follows [22, 23]:

(5) $$\begin{array}{c} Y=\frac{\sum_{i=1}^{n}{\left(g_{i}-g_{i}^{\prime }\right)}^{2}}{n}. \end{array}$$

In equation (5), *n* stands for the number of input samples, *g*_*i*_′ means the model output, and *g*_*i*_ indicates the target output. The mean square error loss function can be obtained by calculating the average variance between the actual model output and the target output. In addition, the cross-entropy loss function is expressed as follows:

(6) $$\begin{array}{c} Y=\frac{1}{n}\sum_{i=1}^{n}\log\left(p_{0}\left(x_{i}\right)\right)+\left(1-g_{i}\right)\log\left(1-p_{0}\left(x_{i}\right)\right). \end{array}$$

In equation (6), *n* and *g*_*i*_ also represent the number of input samples and the target output, respectively; *p*_0_(*x*_*i*_) stands for the model probability output corresponding to *x*_*i*_. Besides, the log-likelihood loss function can be expressed as equation (7):

(7) $$\begin{array}{c} Y=\sum_{i=1}^{n}g_{i}\ln\;p_{0}\left(x_{i}\right). \end{array}$$

The meanings of *n* and *p*_0_(*x*_*i*_) in equation (7) are the same as above.

#### 2.2.2. Examination Methods

The control group was given echocardiography, and the specific examination method included the following steps. Each patient was assisted to select the left decubitus position, and the Philips color Doppler ultrasound diagnostic instrument was used for examination after 15 minutes of quiet state, so as to measure the conditions of left ventricular posterior wall diameter line, interventricular septum, and aorta. Afterward, the blood flow spectrum of the left ventricular of the mitral orifice should be detected, and the change speed of maximum atrial systolic velocity (*A*) and early mitral valve diastolic maximum velocity (*E*) peaks should be measured so that the deceleration time of *E* peak and *E*/*A* value should be calculated. Finally, the blood flow spectrum of aorta and mitral valve can be obtained by measuring the blood flow velocity of the aorta, so the Tei index could be calculated. The deep learning algorithm processing was added to the observation group on this basis.

Since the image is affected by the operation, time, environment, and equipment during the imaging, the final imaging result will have irregular specifications, noise, uneven lighting, and different quality. In order to reduce the interference of these factors on subsequent feature extraction, it is necessary to preprocess the image results. First, binarization threshold segmentation is applied to denoise, and the main process is displayed in Figure 2.

(A) First, the imaging image is converted to a grayscale image, with the size of 99 *∗* 99 mm, the convolution kernel of 33, and the step size of 2.
(B) The between-class variance method is used for binarization threshold segmentation. The specific operation includes the following. The image of target is separated from background, the size of the image *Y (a* *∗* *b)* is set as *a* *∗* *b*, and the initial threshold value is set as *L*. The number of pixels in the pixel set *Y*_1_ whose gray level is below the threshold is *I*_1_, while the number of pixels in the pixel set *Y*_2_ above the threshold is *I*_2_. Besides, the conditions that need to be met are *I*_1_ + *I*_2_ = *a* *∗* *b*. Furthermore, the proportions of *I*_1_ pixel and *I*_2_ pixel are shown in
  (8) $$\begin{array}{c} Q_{1}=\frac{I_{1}}{a*b}, \end{array}$$
  (9) $$\begin{array}{c} Q_{2}=\frac{I_{2}}{a*b}. \end{array}$$

*Y* (*f*, *g*) stands for the pixel value.

The gray value variance between the two types of pixels can be indicated in

(10) $$\begin{array}{c} \Delta \left(Y_{1},Y_{2}\right)=Q_{1}*Q_{2}*\left(t_{1}-t_{2}\right). \end{array}$$

Then, the corrosion operation is employed to remove the surrounding noise blocks to obtain the final binary image.

The image is processed by illumination, in order to balance the overall image brightness and increase the usable data of the model, thereby reducing the interference of subsequent feature extraction. The image light processing method used in this study is the 2D Gamma function method, and its specific calculation process is as follows. First, the image's illuminance-reflection model has to be established.

(11) $$\begin{array}{c} p\left(s,d\right)=h\left(s,d\right)*k\left(s,d\right). \end{array}$$

In equation (11), *h*(*s*, *d*) and *k*(*s*, *d*) stand for the light component and the reflected component in turn, which can reflect the low-frequency and high-frequency characteristics of the image. If the illumination is not uniform, it indicates that the spatial distribution of the *h* component in the image is not uniform, so it needs to be corrected. It is necessary to use the multiscale Gaussian function and the brightness component *P*(*s*, *d*) of the original spatial image to do convolution to extract the illumination component in the image.

In equation (12), *λ* expresses the normalization constant, and *c* represents the scale factor, which can determine the size of the convolution kernel of the Gaussian function. When it is larger, partial global characteristics are extracted; when it is smaller, local characteristics are extracted. Therefore, it is necessary to use unused *c* for synthesis.

Then, the characteristics of the light distribution are adopted to adjust, and the gamma transform is employed to correct.

(12) $$\begin{array}{c} U\left(s,d\right)=255{\left(\frac{P\left(s,d\right)}{255}\right)}^{\gamma }. \end{array}$$

In equation (12), *U*(*s*, *d*) represents the output value, and the enhancement index of brightness can be presented in the following:

(13) $$\begin{array}{c} \gamma =0.5^{1-\left(E\left(s,d\right)/n\right)}. \end{array}$$

In equation (13), *n* indicates the mean value of the illumination component *E*.

### 2.3. Treatment Methods

Patients from the control group were given routine Western medicine treatment. The applied Western medicines included the following. Carvedilol tablets (Cisen Pharmaceutical Co., Ltd.; State Food and Drug Administration (SFDA) approval number: H20113021; specification: 6.25 mg) were taken twice a day, with 3.125 mg each time, and the drug dosage was adjusted according to the patient's tolerance; valsartan tablets (Beijing Novartis Pharmaceutical Co., Ltd.; SFDA approval number: H20173015; specification: 160 mg) were taken once a day, with 80 mg each time; the initial dose of hydrochlorothiazide tablets (Daiichi Sankyo (China) Holdings Co., Ltd.; SFDA approval number: H20100035; specification: 12.5 mg) was 25–100 mg/d, and they were divided into 1-2 times, which could be adjusted according to the patient's condition. Besides, the treatment cycle was 4 weeks. On the basis of the control group, the observation group was given Shengmai injection (Ji'an Yisheng Pharmaceutical Co., Ltd. of Jilin Province; SFDA approval number: Z51022475; specification: 10 mL/bottle). Moreover, the intramuscular injection was adopted once or twice a day (5 mL/time), or intravenous injection could be chosen for 20–60 mL/time, and Shengmai injection was diluted with 250–500 mL of 5% glucose injection, depending on the patient's condition. In addition, 7 days was regarded as a cycle, and the treatment lasts a total of 4 weeks.

### 2.4. Observation Indicators

The hospitalization status of patients from the two groups should be observed and recorded, including the mortality rate, rehospitalization rate, average length of hospitalization, and hospitalization expenses. There was a comparison of the diagnostic accuracy of the two examination methods. Besides, electrocardiogram and echocardiographic parameters as well as patients' quality of life were recorded in both groups at baseline and 5 months after drug treatment. Patients' quality of life was assessed using the SF-36 scale, which consisted of 8 modules. In this study, the focus was on the observation of the general health status, social function, and energy of the patients. The higher the score, the better the quality of life of the patients [24].

### 2.5. Statistical Analysis

The collected data were sorted, summarized, and analyzed by SPSS 23.0. Measurement data were expressed as mean ± standard deviation ($\bar{x}\pm s$), and single sample data were examined by *t*-test. Besides, count data were tested by chi-square, which were represented by (number of cases (%)). In addition,*P* < 0.05 means that the difference is statistically substantial.

## 3. Results

### 3.1. Correction Results of Deep Learning Algorithm

Figure 3 indicates that the processed image was clearer, the light distribution was more uniform, and the visibility was higher.

### 3.2. The Results of Echocardiography in Elderly Patients

The chest radiograph showed that the patient's heart was enlarged markedly. From the echocardiogram on the right side, it was found that the patient's left ventricle was enlarged, so as to oppress the right ventricle (Figure 4). Compared with the heart rate map of the normal population, it revealed that the heart rate of the patients presented sinus tachycardia, which was obviously different from the normal heart rate map (Figure 5).

### 3.3. Rehospitalization Rate and Mortality Rate of Patients from the Two Groups

Table 1 reveals that the rehospitalization rate and mortality rate of patients from the observation group reduced in contrast to those of the control group, but the difference between the two groups was not statistically obvious (*P* > 0.05).

### 3.4. Hospitalization of Patients from the Two Groups

Table 2 indicates that the length of hospitalization and hospitalization expenses of patients from the observation group were lower sharply than those of the control group, with a statistically obvious difference (*P* < 0.05).

### 3.5. Diagnostic Accuracy of the Two Examination Methods

Table 3 reveals that the diagnostic coincidence rate of patients from the observation group was 93.94%, which was higher than 74.29% in the control group, but the difference was not statistically obvious (*P* > 0.05).

### 3.6. Examination Parameters of Patients from the Two Groups at the Basic State and 5 Months after Treatment

Tables 4 and 5 disclose that there was no statistically marked difference in electrocardiographic parameters between the two groups at baseline and 5 months after treatment (*P* > 0.05). However, the echocardiographic parameters at the basic state were compared, finding that only the time of interventricular delay (IVD) of the two groups had a statistically substantial difference (*P* < 0.05). After 5 months of treatment, it was found that the left ventricular electromechanical delay time (LVEMD) parameter value difference between the two groups was statistically remarkable (*P* < 0.05). Furthermore, left ventricular diameter (LAD) and other parameters were compared, showing that there was no significant difference (*P* > 0.05).

### 3.7. Left Heart Diastolic Function of Patients from the Two Groups

Figure 6 suggests that the comprehensive indicator (*E*/*Ea*) and reverse blood flow velocity (*Ar*) of the observation group were lower than those of the control group, while the early and late movement velocity (*Ea*/*Aa*), blood flow velocity (*Vp*), and peak velocity ratio (*S*/*D*) values were higher than those of the control group. Above all, the *E*/*Ea* and *Ar* differences between the two groups were statistically marked (*P* < 0.05).

### 3.8. Quality of Life of Patients from the Two Groups

Table 6 discloses that the quality of life of patients from the two groups improved after treatment, but the observation group was more marked than the control group (*P* < 0.05).

## 4. Discussion

The current clinical methods of diagnosing ALHF can no longer meet the current clinical needs, and the domestic and foreign medical community has proposed echocardiography and other biochemical diagnostic methods [25]. However, there are few related studies now [26]. At present, two-dimensional real-time ultrasound is commonly applied in clinic to evaluate the structure and systolic function of the heart [27]. The examination usually includes the following three steps. The first step is to use the ultrasound probe to scan different positions; the second step is to select the standard section; the third step is to measure and diagnose the determined standard section. After using it, it is found that it has certain limitations, which will be targeted at the section of a specific moment in the cardiac cycle, resulting in poor performance of the final model [28, 29].

In order to improve the diagnostic accuracy of echocardiography and reduce the interference caused by the instability of the imaging results, the deep learning algorithm was used for processing in this study. The results of this study found the specificity, sensitivity, and accuracy of the examination methods of the observation group increased in contrast to those of the control group, suggesting that the diagnosis effect of echocardiography based on deep learning algorithm was better. Currently, there are also studies that proposed the use of N-terminal precursor brain natriuretic peptide (NT-pro BNP) for detection and diagnosis. According to the results of literature studies, it is found that the plasma NT-pro BNP level of elderly patients over 50 years old was higher than 900 pg/mL, while the NT-pro BNP level in elderly patients aged over 75 years exceeds 1,800 pg/mL [30, 31]. In addition, related studies have pointed out that the therapeutic effect of only using the NT-pro BNP detection method to diagnose patients with ALHF does not have a marked impact on the reduction of rehospitalization rate [32]. However, the evaluation and diagnosis applying echocardiography detection method based on deep learning algorithm can reduce the possibility of cardiovascular events in patients with heart failure and decrease the mortality rate and diagnosis and treatment costs [33, 34]. The results of this study also found that the rehospitalization rate and mortality rate of patients in the observation group were lower than those in the control group, which was similar to the related research results [35].

## 5. Conclusion

To sum up, 80 elderly patients with ALHF were selected in this study, and the basic conditions of the patients were first assessed. Then, the different disease assessment and diagnosis methods were used for them, so as to obtain the diagnostic effects of the two diagnostic methods. It was found that the echocardiographic detection method based on deep learning algorithm had a high diagnostic accuracy rate, could reduce the possibility of cardiovascular events in patients with heart failure and decrease the mortality rate and diagnosis and treatment costs, and was worthy of further clinical promotion and use. The shortcoming of this study is that the sample content of the study is small, resulting in incomplete data and deviations in the results of the study. Therefore, the sample size needs to be expanded to further supplement the study to obtain scientific and effective research results, providing reference value for clinical applications.

## Figures and Tables

**Figure 1:** *f*(*x*)/tan*h*(*x*).

**Figure 2:** Denoising flowchart of binarization threshold segmentation.

**Figure 3:** Image correction result (note: the left was the patient's echocardiogram, and the right was the image after the illumination component was corrected).

**Figure 4:** Image examination results.

**Figure 5:** Heart rate chart of the patient.

**Figure 6:** Comparison of left heart diastolic function of all patients.

**Table 1:** Rehospitalization rate and mortality rate of patients from the two groups.

	Number of cases	Rehospitalization rate (%)	Mortality rate (%)
Control group	40	5	6

Observation group	40	3	4

*x*^2^ value		0.039	0.972

*P* value		>0.05	>0.05

**Table 2:** Hospitalization status of patients from the two groups.

	Number of cases	Average length of hospital stay (days)	Average hospitalization cost (ten thousand yuan)
Control group	40	12.3 ± 0.4	1.252 ± 0.06

Observation group	40	8.1 ± 0.7	0.922 ± 0.04

*t* value		0.278	0.236

*P* value		<0.05	<0.05

**Table 3:** The diagnostic accuracy of the two inspection methods.

	Number of cases	Positive	Negative	Coincidence rate (%)
Control group	40	26	14	74.29

Observation group	40	31	9	93.94

**Table 4:** Examination parameters of patients from the two groups at the basic state.

Group	ECG parameters			Echocardiographic parameters			
	Number of cases	Heart rate (beats/min)	PR interval (ms)	QRS time limit (ms)	LAD (mm)	LVEMD (ms)	IVD (ms)
Control group	40	70 ± 12	203 ± 25	173 ± 18	58 ± 22	167 ± 19	60 ± 20

Observation group	40	66 ± 16	193 ± 20	166 ± 12	59 ± 17	160 ± 18	72 ± 10

*P*		>0.05	>0.05	>0.05	>0.05	>0.05	<0.05

**Table 5:** Examination parameters of patients from the two groups after 5 months of treatment.

Group	ECG parameters			Echocardiographic parameters			
	Number of cases	Heart rate (beats/min)	Number of cases	Heart rate (beats/min)	Number of cases	Heart rate (beats/min)	IVD (ms)
Control group	40	71 ± 13	166 ± 15	155 ± 14	54 ± 18	137 ± 24	36 ± 20

Observation group	40	70 ± 14	174 ± 12	144 ± 12	56 ± 22	42 ± 26	37 ± 18

*P*		>0.05	>0.05	>0.05	>0.05	<0.05	>0.05

**Table 6:** Quality of life of patients from the two groups.

		General health condition		Social function		Energy	
Group	Number of cases	Before treatment	After treatment	Before treatment	After treatment	Before treatment	After treatment
Control group	40	52.31 ± 9.21	53.07 ± 8.22	48.11 ± 10.23	56.43 ± 9.41	47.13 ± 9.27	57.33 ± 9.41

Observation group	40	51.26 ± 10.02	66.41 ± 9.24	47.32 ± 10.45	70.73 ± 8.24	46.94 ± 8.26	69.28 ± 9.44

*t* value		0.774	2.274	0.167	4.155	0.058	3.464

*P*		>0.05	<0.05	>0.05	<0.05	>0.05	<0.05

## Data Availability

No data were used to support this study.
